RETRACTED

# Diagnosis of Lumbar Spondylolisthesis Using a Pruned CNN Model

**DOI:** 10.1155/2022/2722315

**Published:** 2022-05-10

**Authors:** Deepika Saravagi, Shweta Agrawal, Manisha Saravagi, Md Habibur Rahman

**Affiliations:** ^1^Department of Computer Application, SAGE University, Indore 452012, India; ^2^IAC, SAGE University, Indore 452012, India; ^3^Physiotherapy Department, Railway Hospital, Kota, Rajasthan 324002, India; ^4^Department of Computer Science and Engineering, Islamic University, Kushtia-7003, Bangladesh

## Abstract

Convolutional neural network (CNN) models have made tremendous progress in the medical domain in recent years. The application of the CNN model is restricted due to a huge number of redundant and unnecessary parameters. In this paper, the weight and unit pruning strategy are used to reduce the complexity of the CNN model so that it can be used on small devices for the diagnosis of lumbar spondylolisthesis. Experimental results reveal that by removing 90% of network load, the unit pruning strategy outperforms weight pruning while achieving 94.12% accuracy. Thus, only 30% (around 850532 out of 3955102) and 10% (around 251512 out of 3955102) of the parameters from each layer contribute to the outcome during weight and neuron pruning, respectively. The proposed pruned model had achieved higher accuracy as compared to the prior model suggested for lumbar spondylolisthesis diagnosis.

## 1. Introduction

A high percentage of the population is affected by lumbar spondylolisthesis. It is a condition in which one of the vertebrae becomes anteriorly misaligned (slips forward) in relation to the vertebrae below it [1–4]. The lumbar vertebra is prone to a variety of developmental defects that can lead to back and neck problems, disabilities, and paralysis [5]. Hence, there is a need to involve technology to diagnose the disease in the early stage before it becomes chronic.

With the advent of Deep Learning (DL), substantial progress has been achieved in automated medical diagnosis [6]. The interdisciplinary collaboration resulted in the development of innovative DL models to investigate spondylolisthesis-related issues, with promising outcomes and substantial potential [7]. As a result, an automated spondylolisthesis diagnosis approach becomes desirable for boosting measuring efficiency substantially [8].

A classification system can help radiologists to enhance their productivity and diagnostic quality. Since public hospitals often have a huge number of patients, this approach will be very valuable for accurate and rapid diagnosis, as well as to avoid long waiting times.  Figure 1 shows some spine X-ray images of normal and spondylolisthesis patients from the dataset.

RETRACTED

Fast diagnosis is the base of the DL model for mobile and small-scale, low-cost devices [9]. But models suggested in prior studies are slow, less accurate, and unsuitable for tiny devices due to a large number of parameters. In this paper, a pruning-based Convolutional Neural Network (CNN) model (i.e., sparse model) is introduced to predict spondylolisthesis in X-ray images early on for fast diagnosis and to avoid chronic situations.

The following are the paper's key contributions:

- A pruned CNN model is proposed for lumbar spondylolisthesis diagnosis which is the first step toward the creation of a lightweight model that can be used on mobile and small-scale, low-cost devices,
- A comparison is made between the weight pruning and unit pruning strategy used in this study,
- The implemented model's accuracy is compared with prior studies given by Azar et al. [10] and Indriana et al. [11]

This paper is organized as follows: (1) Introduction about the need for pruning, (2) Literature Review, (3) Model Architecture, (4) Methodology, (5) Result Analysis and Discussion, and (6) Conclusion.

## 2. Literature Review

Various researchers and practitioners have employed CNNs for pattern classification and function approximations [12–14]. They have utilized the UCI machine learning dataset [15] to categorize the vertebral column diseases using different approaches.

Azar et al. [10] have proposed a pruning-based decision support tool using three different types of decision trees classifiers, Single Decision Tree (SDT), Boosted Decision Tree (BDT), and Decision Tree Forest (DTF), to assist in vertebral column disease diagnosis. The model has achieved a maximum accuracy of 84.84%.

Indriana et al. [11] have ensembled a decision tree (J48) and bagging as the classification model. The model is significant for vertebral disease classification which attains a maximum accuracy of 85%.

Choudhary et al. [16] have used filtered pruning on a CNN model to diagnose breast cancer. The model has achieved 92% accuracy in IDC classification. In [17], the authors suggest a layered pathway evolution approach to compress a Deep Convolutional Neural Network (DCNN) for Digital Breast Tomosynthesis (DBT) mass categorization.

In their study, Hu et al. [18] presented network trimming, which repeatedly optimizes the network by pruning irrelevant neurons based on a big dataset.

Hajabdollahi et al. [19] presented a method for simplifying CNNs using a combination of quantization and pruning. To achieve a simple and efficient network topology, fully connected layers are quantized and convolutional layers are pruned. The simplified network can segment retinal vessels with acceptable accuracy and low complexity.

RETRACTED

In [20], a hierarchical pruning approach is proposed to solve the challenge of decreasing CNN's structural complexity for DR analysis. The original VGG16-Net is used for DR classification after being updated to include fewer parameters. To simplify the network topology, hierarchical pruning gradually removes connections, filter channels, and filters.

In [21], the authors yielded a pruned ANN design that lowered the number of diagnostic variables used during training. Finally, some diagnostic factors in a patient's data record can be eliminated without compromising the accuracy of the diagnosis method.

DiabDeep bypasses the feature extraction stage and acts directly on WMS data in [22], allowing for a more efficient interface for edge devices. Long-short term memory is employed for this purpose. A grow-and-prune training flow is applied which uses gradient-based growth and magnitude-based pruning algorithms to help DiabNNs learn both weights and connections while boosting accuracy and efficiency.

Chen and Zhao [23] have proposed a layer-wise pruning strategy based on feature representation that attempts to reduce complicated CNNs to more compact ones with comparable performance. By eliminating redundant parameters, the suggested technique is capable to reduce the computational cost, and the pruned models achieve equal or even higher performance than the original models.

Han et al. [24] have developed “deep compression,” a three-stage process that combines pruning, trained quantization, and the Huffman coding to minimize the storage requirements of neural networks without compromising their accuracy.

Li et al. [25] proposed an acceleration technique in which filters from CNNs were removed that are recognized as having a little influence on output accuracy. The calculation costs are significantly reduced by deleting filters from the network together with their connected feature maps.

Horry et al. [26] have used internal and external generalization for X-ray based lung cancer diagnosis. In internal generalization, image quality was enhanced, and misclassified images were sent to the prune list for external generalization.

Xiang et al. [27] have introduced a novel pruning approach in which the performance of the model is improved after fine-tuning the model without affecting the model's size.

After a literature survey, we noticed that pruning is an effective strategy for developing a successful and fast model with low computational complexity.  Table 1 illustrates that several researchers have applied multiple pruning methods for specific medical diagnoses. Azar et al. [10] and Indriana et al. [11] worked on vertebral column disease diagnosis, but these models were developed using an MRI dataset (at the advanced stage) and were not suitable for small devices. As a result, a lightweight CNN model for lumbar spondylolisthesis diagnosis with limited training data is presented in this paper.

RETRACTED

## 3. Model Architecture

### 3.1. CNN Model

CNN is a biologically inspired neural network that consists of neurons with learnable weights and biases. It includes several trainable stages, each of which offers a collection of arrays (feature maps) that reflect the extracted information from the input at that stage [28, 29].

Figure 2 shows the simplest CNN model made up of at least one convolutional layer, dense layers, and a SoftMax to calculate the probability distribution for all of the classes investigated. The description of each layer is as follows:

- Convolutional layer: the feature/filter was moved to every available spot on the image in this layer. A feature map is made and places the value of the filter on it. Then, to keep track of the feature, slide the filter over the image, and the result will be sent to the next layer [30]
- Pooling layer: in this layer, the size of the image stack is reduced [27]
- Activation layer: every negative value from the filtered images is replaced by zeros to avoid the values accumulating up to zero, and the transform function activates none only if the input is over a specified number [31]
- Fully connected layer or dense layer: this is the final layer, and the classification takes place here. In this case, we combined filtered and resized images into a single list [32]

In most CNNs, pooling (subsampling) and activation layers are concatenated to the convolutional layers to make them translation invariant and to speed up the training process. By lowering the number of training parameters, the concept of parameter sharing and the local connection is used to make the CNN more computationally efficient. A convolutional layer's stride value, presence or absence of zero-padding, filter size, and the number of channels are all crucial aspects to consider [33].

### 3.2. Pruning Strategy

DL models based on neural networks may be optimized in a variety of ways [34, 35]. One of these improvements is the elimination of connections between neurons and layers, which reduces the overall number of parameters and, therefore, speeds up the processing. Pruning cleans up the CNN by removing unnecessary connections and nodes [36–39].

Pruning approaches start by training a bigger network, then removing weights and nodes that are deemed redundant [31, 40].  Figure 3 illustrates the two approaches used in this study:

- Weight pruning: set the matrix's weights to zero. As seen in Figure 3(a), this relates to removing connections
- Unit/neuron pruning: in unit pruning, the least required neurons were eliminated from the layers. Every neuron in the layer below connects to the layer above; therefore, this necessitates multiplying a large number of floats together. A “sparse” network allows us to skip some of the multiplications by connecting a neuron to only a few other neurons (Figure 3(b))

RETRACTED

## 4. Methodology

For the diagnosis of lumbar spondylolisthesis, a CNN model is built and fine-tuned. The fundamental purpose of training the CNN is to use multiple iterations to obtain the optimal weights. CNN learns from the dataset which is referred to as the network's weight. The performance of the original CNN model is evaluated, and then pruning methods were applied to the model to remove unwanted weights/neurons. The new CNN model (sparse model) is evaluated, and its performance is compared with the unpruned CNN model. The block diagram of the proposed model is shown in Figure 4.

### 4.1. Proposed Model

The customized model is built without using any of the pre-trained network weights to cut down computation time and complexity. Because the image has a large number of pixel values, the network can easily learn the characteristics as the image size reduces.

For analysis purposes, dropout layers, convolutional layers, batch normalization layers, and average pooling layers will be removed. As a result, the model is constructed using REctified Linear Unit (ReLU) activated four hidden layers. These dense layers were fully connected with 1000, 1000, 500, and 200 neurons. For binary classification of disease, the final layer contains 2 neurons. The allocation of tenser in the proposed model is shown in Table 2. The total number of trainable parameters in the model is 3.9 million.

### 4.2. Pruning Algorithm

The application of the CNN model is restricted due to a huge number of redundant and unnecessary parameters. The steps of the pruning algorithm are summarized in Figure 5 and explained in more detail as follows:

Step 1: Train the network to meet a predefined accuracy level by ensuring all successfully categorized input patterns
Step 2: Calculate the associated saliency for each hidden unit
Step 3: Remove the connection between the nodes in two parts:

- Delete the connections between input and hidden nodes
- Then connections between the concealed nodes and output nodes are eliminated

Step 4: Remove units that are less than the desired value
Step 5: Apply the modification to all of the network's weights
Step 6: Compute the prediction performance of the network after retraining it
Step 7: If the performance of the model drops below an acceptance level, then “Stop and revert to the prior network weights setting” Else: “Go to Step 2.”

RETRACTED

### 4.3. Data Collection

The collected radiographs of the vertebrae were classified as normal or spondylolisthesis radiographs by physiotherapy and rehabilitation specialists. The dataset contains spine X-ray images of 337 patients in various diameters. This collection includes 156 images of people with spondylolisthesis and 181 images of normal individuals (without spondylolisthesis).  Table 3 gives a brief description of the dataset used in this study.

### 4.4. Experimental Set-Up

The Google Colab platform was used to build this experiment using Python3 in a windows environment. TensorFlow, a DL framework, is currently at version 2.5.0. The pyplot module from the matplotlib package will then be used to display the accuracy and loss graphs, which provides a MATLAB-like interface to the underlying object-oriented charting library. It creates figures and axes implicitly and automatically to obtain the required plot.

### 4.5. Data Splitting

Using the train_test_split() technique, the dataset is split into two groups in 85 : 15 ratio—the train set (287) and test set (50). The statistics of the split dataset are shown in Table 4.

### 4.6. Training CNN Model

TensorBoard is loaded to monitor the training process, and the model is configured with losses and metrics for model training and performance evaluation. The network is developed to perform a classification task using categorical cross-entropy as a loss function to minimize the loss during model training. All of the tasks are trained end-to-end at the same time using the Adam optimizer. “Adam” is a gradient-based loss function optimization technique that is both simple and computationally efficient having a learning rate of 0.001 (by default). A built-in Keras image data generator is used to generate batches of image data with real-time data augmentation. By eliminating overfitting, data augmentation allows researchers to artificially improve training data.  Table 5 shows the hyperparameters used during the CNN training.

Implemented CNN model is tested for 20 epochs, and metric values are logged into a history object after compilation for tracking progress while training. The accuracy/loss graph is used to demonstrate the metric's ongoing learning. Training accuracy/loss subplots show how the training accuracy/loss (red line) and validation accuracy/losses (blue line) for the models fluctuate as the learning progresses.

Figure 6(a) shows training/validation accuracy, whereas Figure 6(b) shows training/validation loss.

### 4.7. Pruned CNN (Sparse) Model Implementation

TensorFlow's “tensorflow model optimization” module allows pruning. In this experiment, APIs were used throughout the trained CNN model. The pruning technique involves iteratively removing connections between layers, given a sparsity parameter (% of weights eliminated) and scheduling (pruning frequency). A sparsity variable *k* with different percent (i.e., *k* = [0.0, 0.25, 0.5, 0.6, 0.7, 0.8, 0.9, 0.95, 0.97, 0.99]) is used to eliminate weight/neuron from all hidden layers using the formula:

(1) $$\begin{array}{c} {\text{Tensor}}_{\text{size}}-\left({\text{Tensor}}_{\text{size}}\times {\text{sparsity}}_{\text{value}}\right). \end{array}$$

Let the value of the sparsity variable be *k* = 0.25, and the tensor size be 1000; then the total weight reduced at a single layer according to the formula is

(2) $$\begin{array}{c} 1000-\left(1000\times 0.25\right). \end{array}$$

That means 25% of the weight is removed from each layer. The same process is followed for all the sparsity values at each hidden layer. Both weight and unit pruning algorithms used the same sparsity level to reduce the complexity of the model. At last, application programming interfaces (APIs) are used to redefine the network which can be used to change the complete model. After applying sparsity, the accuracy and loss during weight and unit pruning are recorded in Table 6.

RETRACTED

It was noticed during the training process that some hidden nodes of CNN hold a virtually constant output while others vary constantly.  Figure 7 depicts the sparse model's performance during the pruning phase.

In the figure, the blue line shows the training accuracy/loss, and the red line shows the validation accuracy/loss of the sparse model. The dotted curve represents weight pruning on the training data, while the solid curve represents unit pruning.

## 5. Result Analysis and Discussion

The process is started by training a conventional network to learn about connectivity. The training curve for the CNN model is shown in Figure 6. According to that, the accuracy and loss values of the CNN model are 92.12% and 0.79, respectively.

The connections with lower weights are then pruned: all connections with weights less than a specific threshold are removed from the network. After that, the network is retrained to learn the final weights for the sparse links that are remaining.  Figure 7 depicts the sparse model's ongoing learning, which is summarized in Table 6.

The weight pruning approach maintains high accuracy of 94.12% even after trimming 70% of the weights from each layer, after that when we trim the weights further then the model's accuracy declines linearly. However, when the sparsity values increase, we observed that unit pruning outperforms weight pruning as the model's accuracy remains constant under unit pruning even after removing 90% of the neurons from the layers. We have stopped the trimming of weights/neurons when the accuracy of the pruned model starts declining.

RETRACTED

Experimental results reveal that only around 30% (about 850532 out of 3955102) and 10% (about 251512 out of 3955102) of the parameters from each layer contribute to the outcome during weight and neuron pruning, respectively.

The loss represents the match between a prediction and the ground truth label, which decreases over time. The magnitude of weight loss should decrease as the workout progresses. The training loss curve drops more steadily in unit pruning. Weight and unit pruning losses were 0.57 and 0.19, respectively.

The following are the study's unique features:

- The proposed method is the first step toward the creation of a suitable model for lumbar spondylolisthesis diagnosis which can be used on mobile and small-scale, low-cost devices
- Unit pruning strategy is more suitable for this study as it has reduced 90% of the original network's load (more than weight pruning) effectively
- When compared to earlier research suggested by Azar et al. [10] and Indriana et al. [11], the implemented pruned CNN (sparse) model in this work attains a higher accuracy of 94.12%

## 6. Conclusion

CNN has been widely used to solve a variety of issues. In this study, weight and neuron pruning are applied to the CNN classifier. Our finding reveals that there is no decline in accuracy as the sparsity grows from 0 to 70%. This indicates that more than half of the neurons in a neural network are redundant and contribute nothing to the accuracy (the number of redundant neurons is higher in the case of neuron pruning as compared to weight pruning).

Both weight and unit pruning are capable of deleting a sufficient percentage of the network's weight while maintaining accuracy and minimizing loss for initial sparsity values. Implemented sparse model can assist clinicians to diagnose spondylolisthesis through spine X-ray image without sacrificing overall performance. Further study is needed to develop an android application for lumbar spondylolisthesis diagnosis and grading.

## Figures and Tables

**Figure 1:** Lumbar spine X-ray radiographs.

**Figure 2:** CNN model for spondylolisthesis problem.

**Figure 3:** Pruning approaches used in the study.

**Figure 4:** Block diagram of proposed CNN model.

**Figure 5:** Flowchart of implemented CNN pruning process.

**Figure 6:** CNN model's accuracy/loss graph. (a) CNN model's training accuracy. (b) CNN model's training loss.

RETRACTED

**Figure 7:** Sparse model's accuracy/loss graph.

**Table 1:** Summary of literature review.

Source	Purpose	Major findings	Accuracy (%)
Azar et al. [10]	Detection of vertebral column pathology	A decision support tool is proposed for the detection of pathology on the vertebral column using three types of decision trees classifiers.	SDT: 81.94 BDT: 84.84 DTF: 84.19

Indriana et al. [11]	Classification of vertebral column disease	Ensembled decision tree (J48) and bagging are used as the classification model.	Ensemble model: 85% J48: 81%

Choudhary et al. [16]	IDC classification	Pruned models performed superior over original pretrained models.	92.07

Samala et al. [17]	Breast cancer diagnosis	To compress a deep convolutional neural network for mass classification in digital breast tomosynthesis (DBT), a layered pathway evolution strategy is presented.	—

Hu et al. [18]	Network trimming	The zero activation neurons are unnecessary and may be eliminated without impacting the network's overall accuracy.	90.278

Hajabdollahi et al. [19]	Retinal disease screening and diagnosis	A simplification approach is proposed for CNNs based on the combination of quantization and pruning.	76

Hajabdollahi et al. [20]	Detection and analysis of diabetic retinopathy	To simplify the network topology, hierarchical pruning gradually removes connections, filter channels, and filters.	92

Mantzaris et al. [21]	Medical disease prediction	This research uses a genetic algorithm (GA) to prune probabilistic neural networks.	85.5

Yin et al. [22]	Diabetes diagnosis	DiabDeep is a paradigm for widespread diabetes detection that blends efficient neural networks (named DiabNNs) with off-the-shelf WMSs.	94

Chen and Zhao [23]	Reducing complex CNNs	The pruning procedure is conducted at the layer level, and redundant parameters were discovered by studying the features learned in the convolutional layers.	93.03

Han et al. [24]	Deep compression	A three-stage pipeline approach (pruning, trained quantization, and Huffman coding) is introduced to reduce the storage requirement of neural networks.	—

Li et al. [25]	Pruning and compressing	Filters from CNNs that have been recognized as having a little impact on output accuracy have been pruned.	—

Horry et al. [26]	Lung cancer diagnosis	An improved generalization can be achieved with an image preprocessing pipeline that homogenizes and debases chest X-ray images and helps to develop a low-cost, accessible DL system for lung cancer screening.	89

Xiang et al. [27]	Skin disease diagnosis	Without changing the model size, the performance of the model is improved after fine-tuning.	83.5

**Table 2:** Allocation of tensor in proposed CNN Model.

Layer (type)	Output shape	Param No.
Dense_1 (Dense)	(None, 1000)	2353000
Dense_2 (Dense)	(None, 1000)	1001000
Dense_3 (Dense)	(None, 500)	500500
Dense_4 (Dense)	(None, 200)	100200
Dense_5 (Dense)	(None, 2)	402

Total params: 3955102 Trainable params: 3955102 Nontrainable params: 0		

RETRACTED

**Table 3:** Dataset description.

Test cases	337
Normal	181
Spondylolisthesis	156
Image type	X-ray images in .jpg

**Table 4:** Dataset statistics.

Test cases	Train set	Test set	Total
Normal	154	27	181
Spondylolisthesis	133	23	156

Total	287	50	337

**Table 5:** Hyperparameters used while model training.

Hyperparameter	Value
Loss function	categorical_crossentropy
Optimizer	Adam
Learning rate	0.001
Number of epochs	20
Steps per epoch	20
Batch size	16

**Table 6:** Performance of sparse model after applying sparsity.

Index	*k*_sparsity	model_weight	loss_weight	acc_weight	loss_unit	acc_unit
0	0.00	3955102	0.7973	0.9412	0.7973	0.9412
1	0.25	2666327	0.7675	0.9412	0.7751	0.9412
2	0.50	1577552	0.7367	0.9412	0.5957	0.9412
3	0.60	1198042	0.6987	0.9412	0.3913	0.9412
4	0.70	850532	0.5793	0.9412	0.3210	0.9412
5	0.80	535022	0.5641	0.8824	0.1988	0.9412
6	0.90	251512	0.4872	0.8824	0.3407	0.9412
7	0.95	121757	0.3813	0.8824	0.4970	0.7647
8	0.97	72095	0.3723	0.8235	0.6278	0.8235
9	0.99	23713	0.3452	0.8235	0.6467	0.7647

## Data Availability

Access to data is restricted as per patient privacy.
